The article "Antiobesity and Hepatoprotective Effects of Protein Hydrolysates Derived from Protaetia brevitarsis in an Obese Mouse Model" was published in 2022. Journal: Biomed Res Int.

# Antiobesity and Hepatoprotective Effects of Protein Hydrolysates Derived from *Protaetia brevitarsis* in an Obese Mouse Model

**DOI:** 10.1155/2022/4492132

**Published:** 2022-03-27

**Authors:** Eun Hye Lee, So Young Chun, BoHyun Yoon, Man-Hoon Han, Jae-Wook Chung, Yun-Sok Ha, Jun Nyung Lee, Hyun Tae Kim, Dae Hwan Kim, Gyung Yun Beik, Byung Ik Jang, Tae Gyun Kwon, Chae-Eun Park, In-Seon Lee, Bum Soo Kim, Syng-ook Lee

**Affiliations:** ^1^Joint Institute for Regenerative Medicine, Kyungpook National University, Daegu, Republic of Korea; ^2^BioMedical Research Institute, Kyungpook National University Hospital, Daegu, Republic of Korea; ^3^Department of Pathology, School of Medicine, Kyungpook National University, Daegu, Republic of Korea; ^4^Department of Urology, School of Medicine, Kyungpook National University, Daegu, Republic of Korea; ^5^Department of Laboratory Animal Research Support Team, Yeungnam University Medical Center, Daegu, Republic of Korea; ^6^OkChundang Research Institute, Daegu, Republic of Korea; ^7^Department of Internal Medicine, School of Medicine, Yeungnam University, Daegu, Republic of Korea; ^8^Department of Food Science and Technology, Keimyung University, Daegu, Republic of Korea

## Abstract

**Background:**

Obesity induced by excessive nutrients can cause fatty liver and metabolic dysfunction, which leads to hepatic dysfunction and local/systemic inflammatory responses. Previously, we analyzed the antioxidant, antilipotoxicity, and anti-inflammatory effects of protein hydrolysates in vitro. The aim of the present study is to investigate the antiobesity and hepatoprotective effects of protein hydrolysates derived from *Protaectia brevitas* (PHPB) in an obese mouse model.

**Methods:**

For this in vivo study, 40 mice were included and divided into four groups: (1) normal diet group, (2) high-fat-diet (ctrl(–)) group, (3) high-fat-diet and silymarin-treated (ctrl(+)) group, and (4) high-fat-diet and PHPB-treated group. After 6 weeks of treatment, body weight and the amount of daily food intake were observed. Moreover, the major organs and blood of animals were collected for the analysis of serum chemistry, histopathological examination, and obesity- and inflammation-related gene expressions.

**Results:**

The body weight and the amount of daily food intake significantly decreased in the PHPB-treated group compared with those in the ctrl(–) group. The levels of serum ALT, AST, ALP, creatinine, blood urea nitrogen, glucose, bilirubin, total cholesterol, TG, low-density lipoprotein, IL-6, TNF-*α*, and IGF-1 significantly reduced in the PHPB-treated group, whereas the serum free fatty acid, albumin, high-density lipoprotein, and adiponectin concentrations increased. In the analysis of weight of the liver, kidney, lungs, spleen, and fat tissues (from epididymal, perirenal, and mesentery tissues), the PHPB-treated group showed decreased values compared with the ctrl(–) group. In the histopathological analysis, the PHPB-treated group showed significantly reduced macrovesicular fatty change and inflammatory cell infiltration in the liver, and the size of the adipocyte in the epididymis also significantly decreased. The obesity- and inflammation-related gene (IL-6, TNF-*α*, IGF-1, leptin, AP2/FABP4, AMPK-*α*2, *β*3AR, and PPAR-*γ*) expressions in the liver and epididymal adipose tissue were reduced in the PHPB-treated group.

The article "Antiobesity and Hepatoprotective Effects of Protein Hydrolysates Derived from Protaetia brevitarsis in an Obese Mouse Model" was published in 2022. Journal: Biomed Res Int.

**Conclusions:**

Overall, the results of this study suggest that the protein hydrolysates that derived from *Protaectia brevitas* produce antiobesity and hepatoprotective effects via anti-inflammatory activities.

## 1. Introduction

Obesity is an energy overload condition due to excessive calorie intake, which induces systemic metabolic disorders with inflammatory reactions. These disorders manifest as organ dysfunction, and among them, liver dysfunction causes serious effects to the whole body. The obese-related factors that cause liver dysfunction are triglyceride accumulation in the liver, insulin resistance, fatty acid/lipotoxicity, oxidative stress/mitochondrial dysfunction, and inflammation by cytokines/adipokines [1].

The control of inflammatory response can be an effective treatment for the recovery of liver function [2]. Protein hydrolysates (a low-molecular peptide consisting of 3 to 20 amino acids) have various physiological activities, such as antioxidant, antihypertensive, antithrombotic, antiadipogenic, antimicrobial, and anti-inflammatory effects, depending on the composition or sequence [3].

Our team investigated the activities of the protein hydrolysates derived from *Protaectia brevitas* (PHPB) as obtained by five different enzymatic treatments in vitro (alcalase, bromelain, flavourzyme, neutrase, and papain) [4]. Based on the peptide content and SDS-PAGE analyses, PHPB treatment with alcalase or flavourzyme showed a high degree of hydrolysis value. When analyzing the 2,2-diphenyl-1-picrylhydrazyl (DPPH) radical, 2,2′-azino-bis(3-ethylbenzothiazoline-6-sulfonic acid) (ABTS) radical, hydrogen peroxide (H_2_O_2_) scavenging activity, and lipid peroxidation inhibitory activity, the alcalase hydrolysate showed significantly excellent activities. Based on these in vitro experiments, we concluded that the PHPB hydrolysate produces excellent antioxidant, antilipotoxicity, and anti-inflammatory effects.

For the next step, we aimed to investigate the physiological therapeutic effects of PHPB hydrolysate, especially on obesity-induced liver dysfunction via anti-inflammatory effects in an obese animal model. Thus, we analyzed the antiobesity and hepatoprotective effects of PHPB hydrolysate through the analysis of body weight change, food intake, serum biochemistry, target organ/regional fat weight, histopathology, and inflammation-related gene expression in obese mice.

The article "Antiobesity and Hepatoprotective Effects of Protein Hydrolysates Derived from Protaetia brevitarsis in an Obese Mouse Model" was published in 2022. Journal: Biomed Res Int.

## 2. Materials and Methods

This animal experiment was conducted in accordance with the regulations after approval was obtained from the Laboratory Animal Ethics Committee of Yeungnam University (YUMC-AEC2020-040).

### 2.1. Preparation of Protein Hydrolysates

The protein hydrolysates of *Protaectia brevitas* larvae (PBL) were prepared as described previously [4]. Four percent (*w*/*v*) suspension of PBL (Universal Farm's Meal, Sunchang, Korea) powder in distilled water was prepared and heated at 90°C for 20 min, and hydrolysis was performed with the addition of flavourzyme (enzyme to PBL ratio was 1 : 100, *v*/*w*) in a shaking incubator at 100 rpm and 55°C. After 8 h of hydrolysis, the enzymatic reaction was terminated by heating at 90°C for 20 min. The hydrolysates were centrifuged at 13,000 × g for 20 min, and the resulting supernatant was then ultrafiltered using centrifugal filter devices (MWCO, 3 kDa; Amicon Ultra-15, Merck Millipore Ltd., Burlinton, MA, USA) at 5,000 × g for 2 h. The protein hydrolysates with <3 kDa were lyophilized and stored at –80°C for further analyses. The yield of the protein hydrolysate was 39% [4].

### 2.2. Diets and Experimental Design

The experimental animals (6-week-old male C57BL/6J mice) were obtained from Central Lab. Animal Inc. (Seoul, Korea) and adapted to a standard diet (Research Diets, New Brunswick, NJ, USA) for 1 week. The total mice were subdivided into four groups with 10 in each group. They received the following treatment schedule:

1. *Normal*. Normal control mice fed with a standard diet (2.93 kcal/g)
2. *Ctrl(–)*. Mice fed with high-fat diet (rodent diet with 60 kcal% fat, 5.24 kcal/g, D12492, The Jackson Laboratory, Sacramento, CA, USA)
3. *Ctrl(+)*. Mice fed with high-fat diet and treated with silymarin (*GIBCO*-BRL, Waltham, MA, USA) via the gastric gavage route (16 mg/100 g of body weight/daily) for 6 weeks
4. *PHPB*. Mice fed with high-fat diet and treated with PHPB (Okchundang, Daegu, Korea) via the same route (16 mg/100 g of body weight/daily) for 6 weeks

During the experiments, the body weight, food intake, and general symptoms were monitored. The animal husbandry conditions were as follows: polysulfone cage, 200 W × 318 D × 145 H (mm); 5 animals per cage; temperature, 21.0 to 23.3°C; relative humidity, 41.6 to 62.8%; air changes, 10 to 15 clean, fresh, filtered air changes per hour; lighting, 12 hour light/dark cycle, 7 AM to 7 PM via automated timer; intensity of illumination, 150 to 300 Lux; and cage control, cages were replaced once a week, and water bottles were replaced twice a week. Cages and water bottles were washed with an automated washer and sterilized by an autoclave.

The article "Antiobesity and Hepatoprotective Effects of Protein Hydrolysates Derived from Protaetia brevitarsis in an Obese Mouse Model" was published in 2022. Journal: Biomed Res Int.

### 2.3. Blood and Organ Sampling

After an overnight fast, the animals were sacrificed with CO_2_ gas, and the blood and target organs were sampled. The blood collected from the heart was centrifuged at 3,000 rpm for 15 minutes to separate the serum and stored at −80°C until analysis. The extracted liver, kidney, lungs, spleen, and epididymal adipose tissue were weighed; divided into three for histology, RNA, and protein analysis; and stored at −80°C.

### 2.4. Serum Chemistry

The hematological parameters for liver function (alanine transaminase (ALT), aspartate transaminase (AST), alkaline phosphatase (ALP), bilirubin, albumin, glucose), renal function (creatinine, blood urea nitrogen (BUN)), and lipid profiles (total cholesterol (T-chol), triglyceride (TG), high-density lipoprotein (HDL), low-density lipoprotein (LDL), fatty acid) were analyzed using an automatic biochemical analyzer (Hitachi-720, Hitachi Medical, Japan). The inflammatory cytokine/adipokines (*tumor necrosis factor-α* (TNF-*α*), *interleukin 6* (IL-6), leptin, *insulin-like growth factor-1* (IGF-1), adiponectin) were analyzed using enzyme-linked immunosorbent assay (ELISA) kits (R&D Systems, Minneapolis, MN, USA).

### 2.5. Histopathological Examination

The liver and epididymal adipose tissue were fixed in 10% neutral buffered formalin solution, embedded in paraffin wax, cut into 5 *μ*m thick sections, stained with hematoxylin-eosin (H&E), and examined using a light microscope (×200). By a special pathologist, the presence or absence of specific lesions was observed. The adipocyte size of the epididymal adipose tissue was measured using an optical microscope in units of 100 *μ*m.

### 2.6. Analysis of Obesity- and Inflammation-Related Gene Expressions

For the liver tissue, the AP2/FABP4, AMPK-*α*1, AMPK-*α*2, UCP2, leptin, *β*3AR, adiponectin, and PPAR-*γ* mRNA expressions were analyzed using real-time PCR. After the extraction of RNA with RNAsol, cDNA and gene amplification were performed with the One-step SYBR Green PCR kit (Thermo Fisher Scientific) using the Applied Biosystems 7500 Real-Time PCR System (Applied Biosystems, Waltham, MA, USA). The PCR conditions were carried in a cycle of 40 times of reaction at 95°C for 10 seconds and then 5 seconds at 95°C and 30 seconds at 60°C. The product amplified using real-time PCR was quantified using the comparative cycle threshold (Ct) method, and each sample was normalized with the expression level of GAPDH. For the epididymis adipose tissue, the UCP2, leptin, *β*3AR, adiponectin, and PPAR-*γ* mRNA expressions were analyzed using the same method.  Table 1 shows the primer sequences and full name of the genes.

The article "Antiobesity and Hepatoprotective Effects of Protein Hydrolysates Derived from Protaetia brevitarsis in an Obese Mouse Model" was published in 2022. Journal: Biomed Res Int.

### 2.7. Statistical Analysis

The values were expressed as mean ± SD. The analysis of variance and post hoc tests were used to assess the data of the biological activities, with a statistical significance level of *p* < 0.05. The differences in the assay between the treatment and control groups were compared using the unpaired Student's *t*-test.

## 3. Results and Discussion

### 3.1. Effects on Body Weight and Food Intake

At the end of week 10, the body weights of the normal, ctrl(–), ctrl(+), and PHPB-treated groups were 31.97 ± 3.43, 45.89 ± 3.51, 38.61 ± 6.14, and 35.02 ± 3.77 g, respectively (*p* < 0.05) (Figure 1(a)). The rate of weight gain in the normal group was moderate (about 1 g per week), whereas the ctrl(–) group showed about a twofold increase. In the PHPB-treated group, during the first 3 weeks, the body weight increased with the same pattern as the ctrl(–) group, but after PHPB treatment, the weight did not increase after 4 weeks and then increased slowly about 0.5 g/week, which is a pattern similarly observed in the ctrl(+) group. The final weight gain of the normal group was 10.37 ± 2.87 g, ctrl(–) group 20.3 ± 2.0 g, ctrl(+) group 17.31 ± 6.35 g, and PHPB-treated group 13.92 ± 2.99 g, which was a significant decrease compared with the ctrl(–) group (*p* < 0.05) (Figure 1(b)).

The mean intake of the normal diet mice was 152 g (445.36 kcal) in the first week and then gradually increased, and the final was 199 g (583.07 kcal) (*p* < 0.05) (Figures 1(c) and 1(d)). The high-fat-diet (ctrl(–)) group showed a significantly decreased mean intake (135.67 g) (710.91 kcal) on the first week. The mean intake of the ctrl(–) group maintained constantly, and the last mean intake was 136.5 g (715.26 kcal). The ctrl(+) group showed a significant decrease in mean intake at the week of the treatment (green arrow), the low diet was maintained, and the last was 83 g (434.92 kcal). The PHPB-treated group showed a significant decrease in mean intake 1 week after treatment (purple arrow) and then slightly increased, and the last was 118 g (618.32 kcal). Statistically, the dietary of the PHPB-treated group was significantly decreased compared with that of the ctrl(–) group.

### 3.2. Effects on Serum Chemistry

In the analysis of liver function by evaluating the AST, ALT, and ALP in the serum, the PHPB-treated group showed decreased values (790.7 ± 152.2, 112.7 ± 12.4, and 151.6 ± 17.7 U/L, respectively) compared with the ctrl(–) group (818.3 ± 364.0, 164.1 ± 83.7, and 223.8 ± 26.6 U/L, respectively), and a statistically significant decrease in ALP was observed (*p* < 0.05) (Figure 2(a)). In the analysis of renal function by evaluating the creatinine and BUN in the serum, the PHPB-treated group showed relatively decreased values (0.55 ± 0.08 and 27.03 ± 3.04 mg/dL) compared with the ctrl(–) group (0.61 ± 0.11 and 29.43 ± 2.66 mg/dL) (*p* = 0.07 and 0.18) (Figure 2(b)).

The article "Antiobesity and Hepatoprotective Effects of Protein Hydrolysates Derived from Protaetia brevitarsis in an Obese Mouse Model" was published in 2022. Journal: Biomed Res Int.

In the analysis of systemic metabolism and fat conversion to energy by evaluating the glucose, free fatty acid, bilirubin, and albumin in the serum, the PHPB-treated group showed relatively decreased values (68.9 ± 13.3 mg/dL, 65.7 ± 20.1 nM, 000 ± 00 mg/dL, and 1.8 ± 0.1 g/dL, respectively) compared with the ctrl(–) group (125.7 ± 64.7 mg/dL, 45.6 ± 20.9 nM, 000 ± 00 mg/dL, and 1.9 ± 0.1 g/dL, respectively) (*p* = 0.01, 0.04, 0.02, and 0.17) (Figure 2(c)).

In the analysis of lipid metabolism by evaluating the T-chol, TG, HDL, and LDL, the PHPB-treated group showed relatively decreased values in T-chol, TG, and LDL (163.6 ± 14.9, 524.4 ± 49.9, and 11.5 ± 1.6 mg/dL, respectively) and increased values in HDL (90.1 ± 5.4 mg/dL) compared with the ctrl(–) group (189.0 ± 22.7, 575.8 ± 122.8, 14.8 ± 3.3, and 88.2 ± 4.0 mg/dL, respectively) (*p* = 0.0003, 0.23, 0.38, and 0.01) (Figure 2(d)).

In the analysis of inflammatory cytokines/adipokines by evaluating the IL-6, TNF-*α*, IGF-1, leptin, and adiponectin, the PHPB-treated group showed significantly decreased values in IL-6, TNF-*α*, IGF-1, and leptin (19.2 ± 0.6 ng/mL, 253.0 ± 12.1 pg/mL, 24.3 ± 1.2 ng/mL, and 27.67 ± 6.62 ng/mL), but the adiponectin value was relatively increased (85.4 ± 0.8 ng/mL) compared with the ctrl(–) group (21.2 ± 0.8 ng/mL, 316.5 ± 28.7 pg/mL, 27.6 ± 1.0 ng/mL, 35.43 ± 4.48 ng/mL, and 80.3 ± 5.0 ng/mL, respectively) (*p* = 0.0001, 0.0001, 0.0001, 0.006, and 0.005) (Figure 2(e)).

### 3.3. Effects on Target Organs and Regional Fat Weight

In the analysis of the weight changes of the liver, kidney, lungs, spleen, and epididymal (including fat) tissue, the PHPB-treated group showed decreased values (1.33 ± 0.09, 0.43 ± 0.04, 0.20 ± 0.02, 0.06 ± 0.01, and 0.34 ± 0.03 g, respectively) compared with the ctrl(–) group (1.89 ± 0.15, 0.46 ± 0.04, 0.26 ± 0.06, 0.08 ± 0.01, and 0.51 ± 0.05 g, respectively) (*p* = 0.0001, 0.094, 0.005, 0.0003, and 0.0001). The liver and epididymal (including fat) tissue showed a significant decrease in weight (Figure 3).

### 3.4. Effects on the Histopathological Changes

The histopathological changes were observed in the liver (Figure 4(a)). In the normal group, the livers did not show any specific changes in hepatic lobules, sinusoid structures, peri-venous, bile ducts, and portal veins. The hepatocytes showed a cord-shaped arrangement radially toward the edge of the hepatic lobule. The ctrl(–) group showed a fatty liver with a wide distribution of white adipose-accumulating cells, and the Kupffer cells were markedly reduced. Moreover, by pushing the nucleus toward one side of the cell, the macrovesicular fatty change was significantly observed (88%, compared with the normal group) (Figure 4(b)). The infiltration of the inflammatory cells was observed (1.7%%, compared with the normal group) (Figure 4(c)). The liver of the ctrl(+) and PHPB-treated groups showed a significantly reduced range of white adipose-accumulating cells compared with the ctrl(-) group. The macrovesicular fatty change was significantly reduced into 41 and 52%, respectively. Their nuclear morphology showed a distinct appearance similar to that of the normal group. The infiltration of the inflammatory cells also reduced significantly (0.2 and 0.1%, respectively).

The article "Antiobesity and Hepatoprotective Effects of Protein Hydrolysates Derived from Protaetia brevitarsis in an Obese Mouse Model" was published in 2022. Journal: Biomed Res Int.

The adipocyte sizes in the epididymal adipose tissue, which were measured with a unit of 100 *μ*m, in the normal, ctrl(–), ctrl(+), and PHPB-treated groups were 65.99 ± 1.86, 95.94 ± 5.49, 88.14 ± 5.46, and 68.85 ± 5.40 *μ*m, respectively (*p* = 0.0001) (Figure 4(c)). The PHPB-treated group showed a significantly reduced adipocyte size compared with the ctrl(-) group.  Figure 4(d) shows the representative images of the H&E-stained tissues. In the cell shape observation, the normal group showed a homogeneous morphology, whereas the ctrl(–) group showed a heterogeneous morphology. Moreover, the ctrl(+) and PHPB-treated groups showed a relatively reduced heterogeneity compared with the ctrl(-) group.

### 3.5. Effects on Obesity- and Inflammation-Related Gene Expressions

The liver of the PHPB-treated group showed a decreased mRNA expression for AP2/FABP4, AMPK-*α*2, *β*3AR, and PPAR-*γ* (Figure 5(a)), whereas the adiponectin, UCP2, and AMPK-*α*1 expressions were increased compared with the ctrl(–) group (Figure 5(b)). The decrease in AP2/FABP4, AMPK-*α*2, and PPAR-*γ* was significant. For the epididymal adipose tissue, the PHPB-treated group showed a decreased mRNA expression for leptin, *β*3AR, and PPAR-*γ* (Figure 5(c)), whereas the adiponectin and UCP2 expressions increased compared with the ctrl(–) group (Figure 5(d)). The decrease in leptin and PPAR-*γ* and increase in adiponectin were statistically significant.

In this study, we investigated the anti-inflammatory and hepatoprotective effects of PHPB by evaluating the body weight, food intake, serum chemistry, cytokine/adipokine secretion, target organ/epididymal fat weight, histopathology, and expression of obesity-/inflammation-related genes in obese mice.

The article "Antiobesity and Hepatoprotective Effects of Protein Hydrolysates Derived from Protaetia brevitarsis in an Obese Mouse Model" was published in 2022. Journal: Biomed Res Int.

For the body weight, the PHPB-treated group showed only a 1.34-fold increase in weight compared with the normal group and a 2.4-fold increase when compared with the ctrl(–) group, which was a significant weight loss. In the food intake analysis, the average amount of food intake per week significantly decreased in the PHPB-treated group (125.5 g) compared with the ctrl(–) group (145 g). Thus, PHPB seems to induce weight loss and appetite suppression.

For a more specific evaluation of the effects of PHPB, a serum chemistry analysis was performed:

1. The effect on liver was analyzed by evaluating the AST, ALT, and ALP, which are liver synthesis enzymes, and the secretion increased in the fatty liver [5]. Due to the PHPB treatment, the concentration of these enzymes in the blood was reduced, which indicated that PHPB facilitates hepatic function recovery
2. The effect on the kidney was analyzed by evaluating the creatinine and BUN. Creatinine is a metabolite produced by the muscle creatine phosphate, and BUN is urea nitrogen produced via proteolysis [6]. Due to the PHPB treatment, these concentrations were decreased, which indicated the potential renal protective effect of PHPB in obese mice
3. The effect on glucose metabolism was analyzed by evaluating the glucose content. In the PHPB-treated group, the blood glucose level was decreased, indicating that PHPB could affect glucose metabolism leading to the recovery of liver function
4. The effect on fat energy metabolism was analyzed by evaluating the triglyceride value. Triglycerides are energy storage substances, stored in adipocytes, and converted into free fatty acids [7]. The PHPB-treated group showed an increase in triglyceride value, which means that PHPB stimulates fat consumption. In other words, free fatty acid was used as an energy source preferably over glucose. This energy-consuming with triglyceride decomposition influences to inhibition of fatty liver progression and weight loss
5. The bilirubin and albumin concentrations were used as another indicator of liver function. Physiologically, bilirubin binds to albumin, moves toward the liver, enters into the hepatocytes, and excretes to the bile duct [8]. Due to the PHPB treatment, the serum bilirubin concentration was reduced, which indicated that albumin-conjugated bilirubin was excreted easily to the biliary tract, suggesting the recovery of liver function
6. The effect on lipid metabolism was analyzed by evaluating the total serum cholesterol, triglyceride, HDL cholesterol, and LDL cholesterol. In the fatty liver, the lecithin:cholesteric acyltransferase (liver synthesis enzyme) production was insufficient. Thus, the nonesterified cholesterol increased, leading to an increase in the total serum cholesterol levels. The increase in serum triglyceride is related to the lack of lipoprotein lipase (liver synthesis enzyme) [9]. HDL cholesterol removes the excessive cholesterol in the artery, transports to the liver, and discharges out of the body. The PHPB-treated group showed a decrease in the total cholesterol, triglyceride, and LDL cholesterol, whereas HDL cholesterol was increased, which means that PHPB can influence the lipid metabolism in the liver

To investigate the effect of PHPB on cytokine/adipokine secretion, the serum IL-6, TNF-*α*, IGF-1, leptin, and adiponectin content were analyzed. These are representative inflammation-related factors secreted by adipocytes and immune cells. Excessive and ectopic accumulated adipose tissue contains a lot of immune cells, such as macrophages and dendritic cells. As obesity increases, the number of mature immune cells increases, and more inflammatory cytokines are secreted [10]. The abnormally accumulated ectopic adipose tissue also acts like an endocrine organ. The substance secreted by adipocytes is called adipokine, and this mediates the inflammatory response [11]. IL-6 regulates the expression of the *C-reactive protein*, an acute inflammatory reaction substance produced by the liver [12], and transfers information about energy balance from the adipocytes to the hypothalamus [13]. In obesity, the serum IL-6 level is increased. TNF-*α* is synthesized from the adipocytes and stimulates the macrophages, and its expression rapidly increases in obese mice [14]. IGF-1 is derived from the liver, and its activity is increased in obese state [15]. Leptin is produced by the adipocytes and regulates the appetite. In obese cases, leptin concentration is increased [16]. Adiponectin is produced in the adipose tissue and promotes fat oxidation, which acts as an antioxidant [17]. Based on the results of the present study, the PHPB-treated group showed a decrease in the serum IL-6, TNF-*α*, IGF-1, and leptin concentrations, whereas the adiponectin concentration was increased, indicating that the proinflammatory factors were decreased, while the anti-inflammatory factors were increased by the PHPB treatment. Thus, PHPB can function as an inhibitor for systemic inflammation.

The article "Antiobesity and Hepatoprotective Effects of Protein Hydrolysates Derived from Protaetia brevitarsis in an Obese Mouse Model" was published in 2022. Journal: Biomed Res Int.

After systemic analysis, the PHPB effects were focused locally on the target organs. The weight of the liver, kidney, lungs, spleen, and epididymal adipose tissue was reduced in the PHPB-treated group. In obese cases, organ weight change is important, because the increase in organ weight is induced by ectopic fat accumulation. The ectopic fat induces abnormally increased adipokine secretion, resulting in severe inflammation and organ dysfunction [18]. Based on the results of the present study, the PHPB-treated group's organ weight was reduced, particularly in the liver and epididymal adipose tissue. This means that PHPB facilitates the removal of ectopic fat, and it is more effective in the liver and epididymal adipose tissue. The reduction in the weight of the liver and epididymal adipose tissue has an important indication, because the liver is the organ affecting the systemic metabolism and the epididymal adipose tissue is closely associated with the formation of fatty liver [19]. Thus, it is clear that PHPB has a hypolipidemic effect on ectopic fat. This effect was further confirmed through the analysis of histopathology and gene expression.

Based on the histopathological findings, the PHPB-treated liver showed a remarkable reduction in macrovesicular fatty change, inflammatory cell infiltration, and lipid droplets. Thus, the PHPB effect was visualized based on the histopathological changes in the liver, and these changes can be an evidence of functional recovery. Along with this, the adipocyte size in the epididymal fat was measured, which is an important index in obese pathology. Among several fat regions, epididymal fat changes are more important than the others (perirenal, mesenteric, or inguinal region) [19], because inflammatory reaction occurs immediately and severely in the epididymal fat region. Anatomically, the epididymis has not enough space for ectopic fat accumulation [20]. When fat accumulation reaches the maximum volume, inflammatory cell invasion is increased, and this signal promotes inflammatory gene expression [21]. The locally induced inflammation in the epididymis stimulates a systemic inflammatory response, particularly in the liver [19]. Based on our results, the PHPB-treated group showed a significantly reduced epididymal fat volume, and as expected, the proinflammatory gene expression in the epididymis and liver was reduced. Therefore, we confirmed that PHPB induces fat reduction and liver recovery through anti-inflammatory activities.

## 4. Conclusion

In conclusion, we found that the daily oral supplementation of PHPB has systemic effects in terms of weight loss, low appetite, hepatocyte functional recovery, fat metabolism recovery, and anti-inflammation. Also, PHPB has local effects for target organ weight loss, histological liver tissue recovery, size reduction of epididymal adipocyte, and obese- and inflammatory-gene inhibition in the liver and epididymal adipose tissues. Overall, the results of this study suggest the antiobesity and hepatoprotective effects of protein hydrolysates derived from *Protaetia brevitarsis* through anti-inflammatory activities.

The article "Antiobesity and Hepatoprotective Effects of Protein Hydrolysates Derived from Protaetia brevitarsis in an Obese Mouse Model" was published in 2022. Journal: Biomed Res Int.

## Figures and Tables

**Figure 1:** Effects of PHPB on the body weight, food intake, and calories in high-fat diet–induced obese mice. During the experimental period, the body weight (a), final weight gain (b), food intake (c), and calories (d) were measured. The values were expressed as mean ± SD (*N* = 10). Green arrow, a significant decrease in mean value in the ctrl(+) group; purple arrow, a significant decrease in mean value in the PHPB group. Normal: standard diet; ctrl(–): high-fat diet; ctrl(+): high-fat diet with silymarin; PHPB: high-fat diet with protein hydrolysate derived from P. brevitas. Statistically significant value compared with the ctrl(–) group using *t*-test (different letter on the bar means a significance level of *p* < 0.05).

**Figure 2:** Effects of PHPB on the serum biochemistry in high-fat diet–induced obese mice. The indicators for liver function (a), renal function (b), systemic metabolism and fat conversion to energy (c), and adipo-hormones (d) were measured. The values were expressed as mean ± SD (*N* = 10). Normal: standard diet; ctrl(–): high-fat diet; ctrl(+): high-fat diet with silymarin; PHPB: high-fat diet with protein hydrolysate derived from P. brevitas. Statistically significant value compared with the ctrl(–) group using *t*-test (different letter on the bar means a significance *p* < 0.05).

**Figure 3:** Effects of PHPB on the weight of target organs and regional fats in high-fat diet–induced obese mice. The values were expressed as mean ± SD (*N* = 10). Normal: standard diet; ctrl(–): high-fat diet; ctrl(+): high-fat diet with silymarin; PHPB: high-fat diet with protein hydrolysate derived from P. brevitas. Statistically significant value compared with the ctrl(–) group using *t*-test (different letter on the bar means a significance level of *p* < 0.05).

**Figure 4:** Effects of PHPB on the histopathology of the liver and epididymal adipose tissue in high-fat diet–induced obese mice. Representative histological images of the H&E-stained liver tissue at ×200 (a) and ×40 (b) magnification. The adipocyte size (c) and morphology (d) around the epididymis. The values were expressed as mean ± SD (*N* = 10). Normal: standard diet; ctrl(–): high-fat diet; ctrl(+): high-fat diet with silymarin; PHPB: high-fat diet with protein hydrolysate derived from P. brevitas. Statistically significant value compared with the ctrl(–) group using *t*-test (different letter on the bar means a significance level of *p* < 0.05). Scale bars = 100 and 500 *μ*m.

The article "Antiobesity and Hepatoprotective Effects of Protein Hydrolysates Derived from Protaetia brevitarsis in an Obese Mouse Model" was published in 2022. Journal: Biomed Res Int.

**Figure 5:** Effects of PHPB on the obesity- and inflammation-related gene expressions in high-fat diet–induced obese mice. The mRNA expressions in the liver (a, b) and epididymal adipose tissue (c, d) were measured. The values were expressed as mean ± SD (*N* = 10). Normal: standard diet; ctrl(–): high-fat diet; ctrl(+): high-fat diet with silymarin; PHPB: high-fat diet with protein hydrolysate derived from P. brevitas. Statistically significant value compared with the ctrl(–) group using *t*-test (different letter on the bar means a significance level of *p* < 0.05).

**Table 1:** Primer sequences.

Genes	Full name	L	R
AP2/FABP4	Adipocyte protein 2/fatty acid-binding protein 4	5′-tca cct gga aga cag ctc ct-3′	5′-aag ccc act ccc act tct tt-3′
AMPK-*α*2	AMP-activated protein kinase-*α*2	5′-tga gaa cgt cct gct tga tg-3′	5′-ttg ctt ctg ccc ttt cag tt-3′
PPAR-*γ*	Peroxisome proliferator-activated receptor-*γ*	5′-ctg gcc tcc ctg atg aat aa-3′	5′-aat cct tgg ccc tct gag at-3′
Leptin	Leptin	5′-aga tct aca cca ggg acc ct-3′	5-gcc cca cat ttg aga ctg tg-3′
AMPK-*α*1	AMP-activated protein kinase-*α*1	5′-ttg ctt ctg ccc ttt cag tt-3′	5′-agc ata aga agg cag cca aa-3′
UCP2	Uncoupling protein 2	5′-tct tc tggg agg tag cag ga-3′	5′-aca tct gtg gcc ttg aaa cc-3′
*β*3AR	*β*3-Adrenoceptor	5′-aac tct cca acg ctc cag aa-3′	5′-acg gtg aaa ccc att tgg ta-3′
Adiponectin	Adiponectin	5′-gtt gca agc tct cct gtt cc-3′	5′-atc caa cct gca caa gtt cc-3′

## Data Availability

All the data used to support the findings of this study are available in the article.
